This article has been retracted.

# Optimization of Artistic Image Segmentation Algorithm Based on Feed Forward Neural Network under Complex Background Environment

**DOI:** 10.1155/2022/9454344

**Published:** 2022-09-13

**Authors:** Yibiao Li

**Affiliations:** School of Arts and Tourism, Lianyungang Technical College, Lianyungang 222000, China

## Abstract

Based on the theory and application, this paper discusses the optimization of art image segmentation algorithm based on FFNN (Feed Forward Neural Network). In this paper, residual units are used in the corresponding stages of encoder and decoder, and feature information of several convolution layers in each convolution stage of encoder is extracted at the same time. And the feature pyramid module is used to extract multiscale features from the feature map of the last convolution stage in the encoder. Finally, pixel by pixel additions combine the previously mentioned feature information into the corresponding layer of the decoder. Additionally, an improved weight adaptive algorithm based on feature preservation is suggested in this paper, which addresses the issue that the conventional image segmentation algorithm is noise-sensitive. The adaptive connection weight mechanism is also introduced. The accuracy and recall rates of this optimization algorithm can both reach 96.574%, according to the results of 50% cross-validation. All the segmentation performance evaluation indexes of this algorithm are higher than the existing main algorithms. Moreover, the algorithm takes a short time, does not need too much manual intervention, and can effectively segment artistic images. The optimization algorithm in this paper has certain reference significance for the related research of artistic image segmentation.

## 1. Introduction

A significant amount of image data will be produced every day as computer network technology and multimedia technology advance. Additionally, for the purposes of appreciation, communication, and exchange, an increasing number of paintings are being converted into digital images. There is a lot of redundant information in the vast image data. The efficient and accurate extraction of the information from an image has presented significant challenges for computer information processing [1]. These pertinent regions need to be separated and extracted in order to locate and analyze the target, and then the target can be used further [2]. Image segmentation is the process of breaking down an image into various feature primitives [3]. Understanding the content of an image depends on image segmentation, which is crucial in the field of image processing. The outcome of image segmentation directly affects the subsequent operations. Image segmentation is now applicable in a wide range of fields [4]. Its goal is to separate the image into a number of distinct regions, each with their own special characteristics, and then extract the objects of interest. The majority of low-level features used in conventional image segmentation techniques are texture and colour. It is challenging to improve the segmentation effect when the scene is complex or the image contains artefacts. Further research into image segmentation is required because the implementation and application of an efficient image semantic segmentation algorithm has very significant practical implications.

The first and most crucial step in computer vision technology, image segmentation is a key topic in many fields, including image processing [5, 6], pattern recognition [7, 8], and AI. Due to its advantages of independently extracting high-level features from images, NN (Neural Network) has achieved outstanding results in image segmentation tasks in many fields in recent years. A unique deep FFNN is the CNN (Convolutional Neural Network) [9]. The local perception and weight sharing properties of CNN, one of the most widely used deep learning algorithms today, significantly reduce the number of parameters during network training, lowering the risk of over fitting. There are two levels to CNN's basic organisational structure: (1) a layer for feature extraction. The output of the local acceptance domain of the upper layer serves as the input for this layer of neurons, which is used to extract local features from the image. (2) Layer for feature mapping. The neurons on a CNN computing layer consist of multiple feature maps and use the same weight, which helps to reduce parameters and increase efficiency. A convolution layer is connected to a pooling layer in a convolution NN, which typically contains multiple convolution layers and pooling layers. Using the traditional NN to directly perform the full connection operation, although the feature vector of the image can be obtained, with the increase of the complexity of the image digital matrix, the calculated feature vector will be too large, resulting in the inability to carry out subsequent calculations. CNN has a strong feature extraction ability, which can obtain useful information from massive data and complete a number of pattern recognition tasks in image processing [10].

This paper discusses the optimization of art image segmentation algorithm based on forward NN. Its innovations are as follows: (1) in this paper, based on the classical encoder and decoder structure of full convolution NN, aiming at the problem of insufficient semantic information in the high-level stage of the network, we use the large-scale feature extraction ability of void convolution to expand the receptive field of the network, so that the high-level features have more abundant semantic information and make up for the lack of context information. At the same time, aiming at the problem that the image segmented by full convolution network is not fine enough, this paper optimizes the result by modifying the energy function of graph cut algorithm. (2) Aiming at the two shortcomings of traditional image segmentation algorithms, which are the large influence of parameter changes on the segmentation effect and the slow operation speed, this paper analyzes the relationship between image gray difference and suppression weight in image segmentation by introducing new calculation rules of neighborhood weight and neighborhood coupling term and proposes a simplified algorithm based on gray adaptive. At the same time, a multichannel feature fusion module is added to the network decoder to suppress the irrelevant background region response and better recover the details of the image.

## 2. Related Work

Researchers in many fields have always been interested in image segmentation technology, and today many efficient segmentation methods have been proposed. The Boltzmann machine was suggested by Moropoulou and Karoglou to maximise the edge. It derives an iterative conditional mode algorithm from the relationship between images and labels and images and hidden layers to calculate the posterior probability of the target distribution [11]. It simulates the joint distribution of hidden variables and output labels according to input observations. To find and describe local features in images, Eschenfelder et al. proposed an effective scale-invariant feature transformation (SIFT) algorithm. In order to extract their position, scale, and rotation invariants as feature descriptions, it looks for extreme points in the spatial scale [12]. Eschenfelder et al. successfully segmented infrared pedestrians by using the renowned Chan-Vese model to overcome the issues of low signal-to-noise ratio and blurred edges. However, this model's poor capacity for adaptation will result in false segmentation in complex backgrounds [12]. According to Ioannidou et al. and Yuan et al., the NN segmentation method not only takes the characteristics of the image set as a whole into account but also combines the benefits of NN, which has a clear impact on image segmentation [13, 14]. Tajbakhsh et al. proposed a correlation feedback algorithm based on NN from the perspective of machine learning [15]. During the retrieval process, users can mark positive examples similar to the query images and feed them back to the system, and then the system constructs an FFNN and retrieves them again to improve the query results. Al-Milaji et al. proposed a conditional variational automatic encoder. It mainly includes components such as an image encoder that extracts advanced prior from images, a segmentation encoder that extracts advanced prior from segmentation, and a hybrid decoder that outputs segmentation results from advanced prior and input images [16]. Benaichouche et al. used the Otsu algorithm to segment the human body in infrared thermal image, but when the edge of infrared thermal image is blurred and the area is unclear, it will cause serious oversegmentation [17]. The experimental environment adopted by Poudel and Lee is a typical experimental environment with ordinary computing power and research under small data sets [18]. Therefore, it is not necessary to deliberately pursue the unrealistic deep network, but to select the appropriate CNN structure according to the actual environment; the structure may not be complicated, but it is not inefficient. Chiang et al. proposed an edge detection method based on Grossberg-Mingolla model to realize image segmentation. The model reconstructs the image area from the contour line by filling or spreading [19].

In this study, the residual unit is applied to the appropriate encoder and decoder stages, and simultaneous extraction of the characteristic data from multiple convolution layers is performed in each convolution stage. The feature pyramid module is used to extract multiscale features from the encoder's final convolution stage's feature map; after that, the feature data is fused into the corresponding layer of the decoder by adding pixels one at a time. The ability of hole convolution to extract large-scale features is used to increase the network's receptive field at the same time, based on the traditional encoder-decoder structure in full convolution NN, to address the issue of insufficient semantic information in the high-level stage of the network. This will allow the high-level features to have more abundant semantic information and compensate for the absence of context information. This paper optimises the output by altering the energy function of the graph cut algorithm in order to address the issue that the image segmented by a full convolution network is not fine enough. The outcomes demonstrate a notable improvement in the segmentation effect from the suggested algorithm.

## 3. Methodology

### 3.1. Fundamentals of Forward NN Technology

NN is a relatively mature theory in machine learning. Since its development, it has shown certain advantages and potentials in many aspects, especially in the field of pattern recognition, due to its parallel and fault-tolerant characteristics. It can directly find the input-output dependency of the pattern classifier from the training samples. The processing unit in the NN is the simulation of biological neurons, while the directed arc is the simulation of “axon-dendrite” pairs. The interconnection intensity matrix formed by all the comprehensive directed arcs corresponds to the long-term memory of information in the human brain. The processing unit uses nonlinear function to realize the nonlinear mapping between the input and output of the unit, and its instantaneous state value corresponds to the short-term memory of information in the human brain. Presently, an increasing number of people use NN for image processing, particularly image segmentation. The activation function cannot be separated from how the NN operates, and sigmoid function is used in the majority of cases. As a classification problem at its core, image retrieval, the interactive process will be viewed as a training process. The subsequent query process will be classified after users label and categorise the retrieval results. There are two main issues with image retrieval, which are also the focus of this paper's two main research sections. How to effectively extract image features in order to convey the “semantics” of images comes first. The second is how to use the image features that have been extracted and successfully and quickly retrieve the same or similar images. Image segmentation is the technology and procedure for dividing an image into regions with various properties and extracting interesting objects from each region. Here, the target may correspond to a single area or to several areas, and the characteristics may take the form of colour, texture, grayscale, etc. Image segmentation's main goal is to select the best representation of an image so that it can be recognised and understood more easily.

Let the set *R* represent the entire image area, the segmentation of *R* can be regarded as dividing *R* into *N* nonempty subsets *R*_1_, *R*_2_, *R*_3_, ⋯, *R*_*N*_ satisfying the following five conditions:

(1) $$\begin{array}{c} \overset{N}{\underset{i=1}{\cup }}R_{i}=R. \end{array}$$

For all *i* and *j*, *i* ≠ *j*, there are

(2) $$\begin{array}{c} R_{i}\cap R_{j}=\emptyset . \end{array}$$

For *i* = 1, 2, ⋯, *N*, there are

(3) $$\begin{array}{c} P\left(R_{i}\right)=\text{TRUE}. \end{array}$$

For *i* ≠ *j*, there are

(4) $$\begin{array}{c} P\left(R_{i}\cup R_{j}\right)=\text{FALSE}. \end{array}$$

Where *P*(*R*_*i*_) is a logical predicate over all elements in set *R*_*i*_, and ∅ represents the empty set.

The central idea of the traditional feedforward network solution method is to establish the mapping between samples and their categories, but its training method is based on the minimization of a given evaluation function. Its essence is to approximate this mapping by the combination of several functions with predetermined forms and numbers. Feedback technology is a kind of human-computer interaction mechanism technology. The process is that users mark the results retrieved in the previous round. This information is then fed back into the system, which modifies itself in response to it to conduct a new round of inquiry, until the user is satisfied with the results or runs out of patience. Users can use the correlation feedback method to evaluate the results of image retrieval, marking successful images to be fed back into the system for further retrieval for improved outcomes. The forward NN algorithm can categorise the related images and irrelevant images in the feature space into two groups as a result of the user marking the images in the feature space that are close to the query image on a regular basis. As a result, this model can find more related images during subsequent retrieval. Two characteristics of adjacent pixels' pixel values, discontinuity and similarity, can be used to segment an image. The region's pixels are generally similar to one another, but there is some discontinuity at the region's borders. Thus, boundary-based algorithms that use the discontinuity of features between regions and region-based algorithms that use the similarity of features within regions can be used to segment data. Because there is a huge gap between image features and user semantics, and the corresponding relationship is very complex, the improvement of retrieval results by relevance feedback method is limited. However, the correlation feedback technology based on NN assumes that the correlation images conform to the mixed normal distribution in the feature space. Experiments show that the segmentation results of this system can satisfy users more. Image segmentation is a special challenge for the application of NNs. This is partly because the traditional NN lacks the ability to analyze multiple targets at the same time. The two most common network structures, called multilayer perceptron and associative memory, need to store templates or have learning ability first. However, in image segmentation, except those who have prior knowledge, they all need a direct and inherent processing, and the traditional network structure is not competent. This paper improves the network structure.

Every image that the machine “sees” is a digital matrix. In image retrieval and segmentation, the traditional method of feature+distance formula is adopted, and the returned result is the image in the hypersphere with the center of the query image and the radius of a constant in the feature space, as shown in Figure 1.

If A is the query image, the returned results are sorted according to the distance from the image A: A-D-C-B-E-G-F. Because of the diversity of semantically similar images, the distribution of these images in the feature space is diverse, and it is difficult to describe them with some standardized geometric shapes. The combination of NN and image-related feedback is a hot research topic in recent years. It assumes that there is a nonlinear relationship between the features of images, and the feedback samples of users are used as training samples of NN. Through the learning of NN, the performance of the system can be further improved. Because NNs can be quickly applied to classification, they are applied to image segmentation based on pixel classification. Because the correlation of time provides a good way to represent different targets in NNs, many NNs used in image segmentation revolve around this center. At present, the basic image segmentation is divided into threshold segmentation, region segmentation, edge segmentation, and segmentation based on energy functional. These segmentation methods mainly use the characteristics of digital images to complete the segmentation process. The principle and implementation details are relatively simple, and the algorithm performance is relatively stable. Threshold method is the simplest image segmentation method. These methods divide the image pixels according to their intensity levels. The process of region segmentation involves breaking the original image into a number of smaller regions, merging pixels with related properties to create the target region, and then cutting the target region into a number of smaller regions. The idea behind edge-based segmentation is to divide an image into smaller pieces by identifying the contour of the target edge. Filtering, enhancement, detection, and location can be roughly classified as parts of the process.

### 3.2. Optimization of Art Image Segmentation Algorithm Based on NN

Due to the weight sharing ability of convolution operation, different features in the image can be extracted by convolution kernel with the same weight on the image. Therefore, compared with fully connected network, CNN parameters are better. The working principle of convolution kernel is to divide the image into a small piece, usually called receptive field, which is helpful to extract the feature map. In standard CNN, after many pooling operations, the resolution of the feature map will be rapidly reduced, resulting in the loss of the spatial structure information of the original image, which will have a certain impact on image semantic segmentation. Void convolution makes up for this defect, so that the characteristic map output by each convolution layer contains a wider range of information. Each neuron in each row of the network adjusts its weight through fuzzy competitive learning until the network converges to the minimization of the energy function. At this time, the state of the network is the result of grayscale fuzzy clustering. Mapping this result back to the image space, we can get the image segmentation result. The decoding operation of the model is completed by deconvolution and depooling, so the pooling operation of the model does not retain the maximum pooled index value, and the spatial location relationship of aggregation features is not introduced in this process. This operation can restore the aggregated feature to the corresponding position according to the pooled index value, and through convolution encryption with a learnable convolution kernel, the obtained new feature map contains rich position information.

The feature pattern produced by the convolution operation can appear throughout the image in various locations. It is no longer necessary to know a feature's precise position after it has been extracted using a convolution layer as long as its approximate position in relation to other features is preserved. Downsampling or pooling is a crucial local operation. It compiles comparable data close to the receptive field and produces the dominant response in this locality. The convolution network will use the upsampling operation to enlarge the image until the original image size in order to achieve the classification of the pixels in the original image. The upsampled image is the final result, and every pixel in the output image can then be predicted. The approach is to calculate the probability—or maximum value of the image pixel at this location in all final images—and then rank each category according to that probability. In this study, the input layers of the generator and discriminator, respectively, each receive conditional variables. The conditional generation confrontation network transforms into an image segmentation model when the conditional variables are the pixel-level labels of images, and it is able to produce segmentation results with better continuity in pixel space after training. In batch normalisation, the input of any layer is set to the standard normal distribution of zero mean and unit variance through a series of normalisation operations. The gradient can be preserved by adjusting the data distribution, which is typically done before the convolution layer in CNNs. Additionally, it can quicken network learning and smooth the gradient, which will aid in enhancing the network's generalisation capabilities.

First of all, the average value of data in a small batch is required:

(5) $$\begin{array}{c} u_{B}=\frac{1}{m}\overset{m}{\underset{i=1}{\sum }}x_{i}. \end{array}$$

*m* is the number of batches in the stochastic gradient descent algorithm. Then you need to find the variance of the small batch of data:

(6) $$\begin{array}{c} \sigma_{B}^{2}=\frac{1}{m}\overset{m}{\underset{i=1}{\sum }}{\left(x_{i}-u_{B}\right)}^{2}. \end{array}$$

Perform a normalisation operation on each element in the batch:

(7) $$\begin{array}{c} {\hat{x}}_{i}=\frac{x_{i}-u_{B}}{\sqrt{\sigma_{B}^{2}+\int }}. \end{array}$$

Finally, scale and offset operations are performed to transform the data back to the original distribution:

(8) $$\begin{array}{c} {\text{BN}}_{\gamma ,\beta \left(x_{i}\right)}=\gamma {\hat{x}}_{i}+\beta . \end{array}$$

Among them, *γ* and *β* are two trainable parameters. Consider an image containing multiple regions *R*_1_, *R*_2_, ⋯, *R*_*q*_, assuming that inside each region, the image can be represented as a white noise driven autoregressive model. Let the image of region *R*_*i*_ be represented by the *k*_*i*_-th class model, and the point probability density function of this region is *P*_*k*_*i*__(*x*_*R*_*i*__), and *x*_*R*_*i*__ is the point set of the region.

Since points falling in disjoint regions are generated by different linear filters, these points are independent of each other, and for a given region good, with *R*_1_, *R*_2_, ⋯, *R*_*q*_, the probability density of all *x* in the image is defined as

(9) $$\begin{array}{c} p\left(x\left|R_{1},R_{2},\cdots ,R_{q}\right.\right)=p_{k_{1}}\left(x_{R_{1}}\right)p_{k_{2}}\left(x_{R_{2}}\right)\cdots p_{k_{q}}\left(x_{R_{q}}\right). \end{array}$$

The logarithmic form of the display expression of the density function obtained from the linear prediction error residual of each image model is

(10) $$\begin{array}{c} -2\ln p\left(\hat{x}\left|R_{1},R_{2},\cdots R_{q}\right.\right)=\overset{q}{\underset{i=1}{\sum }}\underset{R_{i}}{\sum }\left[\frac{{\left(w_{n,m}^{k_{i}}\right)}^{2}}{{\left(\sigma_{k_{i}}\right)}^{2}}+\ln{\left(\sigma_{k_{i}}\right)}^{2}\right]+\text{NM}\ln2\pi . \end{array}$$

Where $\hat{x}$ is the observation data vector, *w*_*n*,*m*_^*k*_*i*_^ is the error residual calculated by the *k* class filter, and (*σ*_*k*_*i*__)^2^ is the white noise variance of class *k*.

Deconvolution or bilinear interpolation can resize the reduced feature map to its original size, but they are unable to fully replace the lost information, leaving the model's segmented object with blurry edges and incomplete details. This paper addresses these issues by fusing the feature information of convolution NN at all levels, resulting in richer low-level and high-level features that support image segmentation and lessen the impact of information loss brought on by repeated pooling and convolution operations on segmentation outcomes. The graph cutting algorithm is also improved in this paper by changing the energy function. First, the probability graph's expression is modified and converted to polar coordinates for calculation. The energy function is then added to the probability term for each pixel in this segmentation result. After numerous iterations, the correct ratio of each function term is determined, resulting in the creation of an optimised boundary curve. Finally, it is mapped to the original image, and a clear boundary of the image is obtained. The structure diagram of CNN is shown in Figure 2.

The following describes CNN's training optimization process: (1) the input image is propagated forward through the path of the input layer, hidden layer, and output layer in order to obtain the output value after the network weight has been initialised. (2) Determine the discrepancy between the forward propagation output result and the desired outcome, and then train the network repeatedly by varying parameters like the offset term and network weight to maximise the forward propagation output value. (3) Send the error back to the network when it exceeds the expected value by computing the error at each layer in turn to determine the network's overall error. The decoder's job is to upsample the encoder's low-resolution feature map using pixel interpolation or transpose convolution and map the features to the full-resolution output prediction feature map for the purpose of pixel classification. The classification of pixels at the pixel level is necessary for image segmentation. It is necessary to combine a multilayer decoder structure to perform upsampling in this process because the feature image output by the encoder is frequently shaky and a significant amount of spatial position information is lost. This allows the accurate boundary information of the object to be recovered. In this study, channel splicing is used to cascade the convolution features of the encoder and decoder in the corresponding stages, which are then sent to a new convolution layer for additional analysis and category prediction. In order to achieve precise segmentation results, the model can fully utilise the features acquired at each level of the coding-decoding network thanks to the concept of cascaded multilevel features.

## 4. Result Analysis and Discussion

The experiment in this section is carried out on the image database Painting-91. There are 2,336 art paintings by 50 painters in the image database, which are divided into portraits, landscapes, scenes, etc. according to their contents, and 13 schools such as constructivism, cubism, impressionism, and popism according to their schools. When organizing the image database according to the visual information, the image features do not distinguish artists, so different artists of the same genre are not distinguished. In all marked images, 3000 images are randomly selected as the training set and 800 images as the verification set. The experimental environment of this paper is carried out on its own server, and the configuration of software and hardware environment required for the experiment is shown in Table 1. All the experimental training is carried out in the GPU environment. As the convolution network increases in depth and level, and the number of neuron nodes increases, it will have high requirements on hardware, and the hardware here is mainly GPU.

The number of images can be multiplied by several times after using image enhancement technology. This paper uses image flipping, image mirroring, and image blurring as image enhancement techniques. Additionally, the artwork image itself is more complex because the data set is a small-scale data set and the experimental environment also uses standard computing power. This paper first normalises the training set and verification set to 256256 to enhance the CNN training efficiency and ease the experimental procedure. Second, each image is rotated by 90, 180, and 270 degrees, respectively. Third, each image is vertically and horizontally mirrored. Random gradient descent is used to optimise the training process. The main training parameters and the required time are shown in Table 2.

In the algorithm, the training part is used to complete the construction of the algorithm network model. In the process of training, different values are given to the parameters to obtain different results, and then the test set is used to record and analyze the results of the network model. The training results of different networks are shown in Figure 3.

Among them, the lower the loss value, the better the trained NN. It can be seen that the network in this paper has achieved good experimental results.

In this section, four evaluation metrics are used to evaluate the performance of the algorithm, namely, accuracy rate (*P*); recall rate (*R*); *F*_*β*_ index (*F*_*β*_); and *J* index (*J*). The definitions of each index are as follows:

(11) $$\begin{array}{c} P=\frac{S_{1}}{S_{2}}\%, \end{array}$$

(12) $$\begin{array}{c} R=\frac{S_{1}}{S_{3}}\%, \end{array}$$

(13) $$\begin{array}{c} F_{\beta }=\frac{\left(1+\beta^{2}\right)PR}{\left(\beta^{2}P+R\right)}, \end{array}$$

(14) $$\begin{array}{c} J\left(S_{1},S_{3}\right)=\frac{\left|S_{1}\cap S_{3}\right|}{\left|S_{1}\cup S_{3}\right|}. \end{array}$$

In the formula, *S*_1_ represents the set of correct pixel points extracted by the algorithm, *S*_2_ represents the set of all pixel points extracted by the algorithm, and *S*_3_ represents the set of all pixel points in the marked area in the label.

The *F*_*β*_ index is the average of the weighted reconciliation of recall and accuracy, and the closer the *F*_1_ index is to 1, the better the segmentation effect. The *J* index is used to measure the regional similarity between the segmentation results of each algorithm and the manual segmentation results. The closer the *J* index is to 1, the better the segmentation effect.

The segmentation performance of this algorithm is compared with the Otsu algorithm and Chan-Vese algorithm, respectively. The accuracy test results of different algorithms are shown in Figure 4. The recall test results of different algorithms are shown in Figure 5.

This algorithm has high levels of accuracy and recall, as can be seen. The advantages of this algorithm include its ease of use, outstanding performance, accurate boundary extraction, and good object contour extraction. One of them, the Chan-Vese algorithm, requires gradient information during segmentation, and the noise in the original signal's influence will lead to numerous false local minima in the gradient map, resulting in oversegmentation.  Figure 6 illustrates the outcomes of various algorithms' *F*_1_ tests. In Figure 7, various algorithms' *J*-index test outcomes are displayed.

One can draw the conclusion that this model performs better overall than the comparison model. This demonstrates in full how this paper's integration of features at various levels can add more context information to the final prediction, and it also demonstrates how well the model performs generally. The comparison results of the number of segmented regions of different algorithms are shown in Table 3.

Generally speaking, the algorithm in this paper is more adaptable to images, and its segmentation effect is better than other common image segmentation algorithms and the traditional legend lateral model algorithm. However, in contrast, in order to remove noise and obtain more image details, the adaptive league algorithm based on feature preserving weights has higher computational complexity.

Cross-validation is a method to evaluate the performance of predictive model classifier. Its purpose is to train a stable model. This training method can effectively avoid overfitting and underfitting. N-fold cross verification means that the original data set is equally divided into N groups, each group of subdata sets is verified once, and the remaining N-1 subsets are used as training sets to participate in the training optimization of the network. Finally, based on this batch of data, N models are trained, and the average prediction accuracy of N models is taken as the final evaluation index of the models. The results of this algorithm's 50% cross-validation segmentation on the test set are shown in Table 4.

In this study, the last three stages of the encoder and decoder's convolution features are added to and fused pixel by pixel using jumping connections before being concatenated. In addition, the hierarchical dependence of features extracted by deeper convolution layers is taken into consideration, which maintains the local consistency of features and enhances segmentation performance. On the one hand, it can reduce the complexity of the model after cascading multilevel features and make the network training process simpler. The experimental results in this section show that the accuracy rate of this optimization algorithm can reach 96.574%, and the recall rate can reach 97.053%. Compared with other models, this model obviously improves the segmentation effect. It has certain reliability and practical significance to apply the optimization algorithm in art image segmentation.

## 5. Conclusion

Pattern recognition, image processing, image editing, and other fields frequently use image segmentation, which is a crucial component of image processing. It connects the various threads of the entire investigation. It serves as both a basis for further image analysis and interpretation and a test of all image preprocessing effects. If users of digital artistic images lack sufficient artistic knowledge, it can be very challenging for them to accurately describe images with semantic tags. This paper discusses the enhancement of the art image segmentation algorithm using FFNN. The traditional image segmentation algorithm in this paper has two drawbacks: the operation speed is slow and the parameter change has a significant impact on the segmentation effect. The relationship between image grayscale difference and suppression weight in image segmentation is analyzed by introducing a new calculation rule of neighborhood weight and neighborhood coupling term, and a straightforward algorithm based on grayscale self-adaptation is proposed. A multichannel feature fusion module is simultaneously added to the network decoder section to suppress the response of irrelevant background areas and improve the recovery of the image's detailed information. This paper optimises the outcome by changing the energy function of the graph cutting algorithm in order to address the issue that the image segmented by the full convolution network is not fine enough. A comparison of the algorithm used in this paper with other image segmentation algorithms is made before the experimental outcomes of creative image segmentation are presented. According to the experimental findings, this optimization algorithm's accuracy can reach 96.574%, and its recall rate can reach 97.053%. Evidently, this model improves the segmentation effect when compared to other models. New feature fusion techniques or paths may be taken into account in the future to lower the weight scale and boost the model's segmentation precision and training effectiveness.

## Figures and Tables

**Figure 1:** Schematic diagram of the constructive learning algorithm.

**Figure 2:** Schematic diagram of CNN structure.

**Figure 3:** Main parameters and training time.

**Figure 4:** Accuracy test results of different algorithms.

**Figure 5:** Recall test results of different algorithms.

**Figure 6:** *F*_1_ test results of different algorithms.

**Figure 7:** *J*-index test results of different algorithms.

**Table 1:** Software and hardware environment configuration.

Deploy	Parameter
Processor	Intel® Core™
Internal storage	8GB
Display card	NVIDIA GeForce GTX 1080
Operating system	Windows, Ubuntu
Exploitation environment	MATLAB, Microsoft visual studio community
Deep learning framework	PyTorch

**Table 2:** Main parameters and training time.

Main parameter	Numerical value
Learning rate	0.0001
Momentum	0.98
Weight attenuation	0.0002
Maximum number of iterations	10000
Training duration	8 h

**Table 3:** Comparison of the number of divided regions.

Segmentation method	Original image	LEGION lateral	Adaptive LEGION	Otsu threshold	Watershed method	Paper method
Number of regions	92	95	94	87	310	93
Effective area	92	92	92	87	85	92
Lost area	/	0	0	6	0	0
Oversplitting	/	3	1	0	246	1

**Table 4:** The cross-validation results of the algorithm in this paper.

Number of experiments	*P*	*R*	*F*	*J*
1	96.012%	96.589%	0.954	0.917
2	96.574%	96.391%	0.947	0948
3	95.894%	97.046%	0.958	0.956
4	96.371%	97.053%	0.939	0.938
5	96.518%	96.982%	0.956	0.965

## Data Availability

The dataset used to support the findings of this study are available from the corresponding author upon request.
